The article "MiR-26a and miR-144 inhibit proliferation and metastasis of esophageal squamous cell cancer by inhibiting cyclooxygenase-2" was retracted in 2026. Reasons: duplicated images; original data or images not available.

# MiR-26a and miR-144 inhibit proliferation and metastasis of esophageal squamous cell cancer by inhibiting cyclooxygenase-2

**DOI:** 10.18632/oncotarget.7908

**Published:** 2016-03-04

**Authors:** Ying Shao, Peng Li, Sheng-Tao Zhu, Ji-Ping Yue, Xiao-Jun Ji, Dan Ma, Li Wang, Yong-Jun Wang, Ye Zong, Yong-Dong Wu, Shu-Tian Zhang

**Affiliations:** ^1^ Department of Gastroenterology, Beijing Friendship Hospital, Capital Medical University, National Clinical Research Center for Digestive Disease, Beijing Key Laboratory for Precancerous Lesion of Digestive Diseases, Beijing, China; ^2^ Department of Critical Care Medicine, Beijing Friendship Hospital, Capital Medical University, Beijing, China

**Keywords:** cyclooxygenase-2, esophageal squamous cell cancer, proliferation and metastasis, miR-26a, miR-144

## Abstract

The altered expression of miRNAs is involved in carcinogenesis of esophageal squamous cell carcinoma (ESCC), but whether miRNAs regulate COX-2 expression in ESCC is not clear. To this end, the expression levels of miR-26a and miR-144 in ESCC clinical tissues and cell lines were investigated by qRT-PCR. COX-2 and PEG2 were quantified by western blot and ELISA. Decrease in miR-26a and miR-144 expression in ESCC was found by a comparison between 30 pairs of ESCC tumor and adjacent normal tissues as well as in 11 ESCC cell lines (*P* < 0.001). Co-transfection of miR-26a and miR-144 in ESCC cell lines more significantly suppressed cell proliferation, migration, and invasion than did either miR-26a or miR-144 alone (all *P* < 0.001), as shown by assays of CCK8, migration and invasion and flow cytometry. The inhibitory effect of these two miRNAs *in vivo* was also verified in nude mice xenograft models. COX-2 was confirmed as a target of miR-26a and miR-144. In conclusion, miR-26a and miR-144 expression is downregulated in ESCC. Co-expression of miR-26a and miR-144 in ESCC cells resulted in inhibition of proliferation and metastasis *in vitro* and *in vivo*, suggesting that targeting COX-2 may be the mechanism of these two miRNAs.

## INTRODUCTION

Esophageal carcinoma is the eighth most common cancer worldwide and the sixth leading cause of cancer death [1]. Esophageal squamous cell carcinoma (ESCC) is a common type of esophageal cancer in China—about 210 000 patients die each year of ESCC, or 52% of all ESCC deaths worldwide [2]. Because ESCC is frequently diagnosed at the advanced stages of disease, the overall 5-year survival rate is less than 15% [3]. Therefore, it is important to delineate the potential mechanisms of tumor development, to find novel therapeutic targets for ESCC.

Cyclooxygenases 1 and 2 (COX-1 and COX-2) are the rate-limiting enzymes involved in the biosynthesis of prostaglandins. COX-1 is constitutively expressed in most tissues, while COX-2 is the inducible isoform, which is responsible for the elevated production of prostaglandins in response to various inflammatory stimuli, hormones, and growth factors [4]. Accumulating evidence supports that COX-2 is involved in both tumor development and progression [5–10], including ESCC [11–16]. It has been reported that aspirin and other nonsteroidal anti-inflammatory drugs are protective against ESCC and adenocarcinoma [17]. We and others have shown that (i) COX-2 expression is a frequent phenomenon in human ESCC tissue samples and positive expression is related with lymphatic metastasis [16, 18–22], (ii) COX-2 inhibitors can inhibit tumor cell proliferation and induce apoptosis by inducing G0 / G1 cell cycle arrest and suppressing Bcl-2 expression [15, 23] as well as prevent tumor formation *in vivo* through the inhibition of COX-2 [14]. (iii) COX-2 inhibitors also inhibit migration and invasion of ESCC cells [24]. Therefore, COX-2 is an important therapeutic target for ESCC treatment.

Presently, there are three main approaches to block COX-2: COX-2 inhibitors, inhibitive transcription factors and post-transcriptional control. The application of the first two methods is restricted, because of the adverse reaction to COX-2 inhibitors [25–26] and the non-specificity of transcription factors. MicroRNAs (miRNAs), a family of endogenous, small non-coding RNAs (20-25 nucleotides in length), are important regulators in a variety of biological processes, including cell development, infection, immunity, and carcinogenesis, through post-transcriptional regulation of mRNA expression. MiRNAs can be classified as either oncogenes or tumor suppressors. Currently, miRNAs have been used in clinic for predicting cancer classification, prognosis, and response to therapy [27–29]. Regulation of COX-2 expression by miRNAs has been extensively studied in a variety of human tumors, but this kind of regulation in ESCC remains unclear [30–40].

We searched the databases TargetScan, PicTar, miRwalk, DIANAmT, microRNA, Microcosm Targets and MicroRanda for miRNAs that might bind to the 3′ -UTR of COX-2. Four candidates including miR-101, miR143, miR-26a and miR-144 were found via computational prediction of microRNA targets. In our preliminary experiments to examine the effect of those 4 miRNAs on proliferation function of ESCC cell lines, we found that miR-101 or miR-143 could inhibit the proliferation of ESCC cell lines, but miR-26a or miR-144 alone did not. In addition, we have reported that miR-101 inhibits ESCC proliferation and metastasis by regulating COX2 [41]. However, Guo et al. found that miR-26a and miR-144 were associated with the different tumor stage classifications (Table 1 in the reference paper [42]) [42]. Therefore, we hypothesized that both miR-26a and miR-144 could inhibit ESCC by inhibiting COX-2.

**Table 1:** The percentage of cells in different cell cycle phases

		G0+G1	S	G2+M
EC9706	Parent	57.1 ± 1.3	31 ± 2.1	12.0 ± 0.9
	Vector	58.2 ± 1.1	30 ± 2.3	12.0 ± 1.1
	MiR-26a-144	66.9 ± 1.2 *	25 ± 1.1	8.1 ± 0.7
EC109	Parent	47.5 ± 1.3	37.9 ± 2.4	11.4 ± 0.9
	Vector	46.7 ± 1.1	50.3 ± 2.3	1.4 ± 0.6
	MiR-26a-144	54.3 ± 1.1 **	30.2 ± 1.1	12.3 ± 0.5

* *P* < 0.001;

** *P* < 0.01 compared with the parent cells and vector-control cells.

In this study, we focused on the potential roles of miR-26a and miR-144 in ESCC development. We examined the expression levels of miR-26a and miR-144 in tumor tissue specimens and cell lines of human ESCC; evaluated the effects of both miR-26a and miR-144 on ESCC cell proliferation, migration, and invasion through *in vitro* assays; and examined the anti-tumor activity of both miR-26a and miR-144 *in vivo* in a xenograft nude mouse model of ESCC. Our study showed that miR-26a and miR-144 inhibit proliferation and metastasis of ESCC by inhibiting COX-2 expression. This may be the first report of miR-144 / COX-2 pathway in human cancer.

## RESULTS

### MiR-26a and miR-144 are frequently downregulated in human ESCC tissues and cell lines

The expressions of miR-26a and miR-144 in clinical specimens of ESCC and corresponding adjacent normal tissues obtained from 30 patients with ESCC. Compared to adjacent normal tissues, the expressions of miR-26a and miR-144 were significantly downregulated in tumor tissues (Figure 1A, 1B). The expression levels of miR-26a and miR-144 in 11 ESCC cell lines were also significantly lower compared with that of Het-1A, a human immortalized esophageal epithelia cell line (Figure 1C, 1D).

**Figure 1:** Downregulation of miR-26a and miR-144 in human ESCC tissues and cell lines The expression levels of miR-26a **A.** and miR-144 **B.** in 30 pairs of ESCC tumor tissues and corresponding normal tissues were determined by quantitative real time RT-PCR as described in Materials and Methods. The expression levels of miR-26a **C.** and miR-144 **D.** in eleven ESCC cell lines and a human immortalized esophageal squamous cell line (Het-1A) were also quantified. Results were calculated by 2^−ΔΔCT^ method and shown as the mean value of three independent experiments. U6 was used as an internal control for data normalization of RT-PCR. Columns and error bars represent standard deviations from three independent measurements. ** *P* < 0.01; *** *P* < 0.001.

### Co-expression of miR-26a and miR-144 cooperate to inhibit the proliferation of ESCC cells

To investigate the biological function of miR-26a and miR-144 in ESCC, we examined the proliferation of ESCC cells. CCK8 assay data showed that proliferation of EC9706 and EC109 cell lines stably transfected with miR-26a or miR-144 was not inhibited, while the percentage of growth inhibition in co-expressed miR-26a and miR-144 was significantly inhibited (Figure 2A).

**Figure 2:** Co-transfection of both miR-26a and miR-144 inhibited the proliferation of ESCC cells **A.** Cell proliferation potentials or growth curves of the cells stably transfected with single miRNA or both of them were determined by CCK-8 assay. Growth curve was generated, according to the absorbance value at different time points (left panel for EC9706 and right one for EC109 cells). **B** and **C.** After 24-h culture, medium was replaced by fresh serum-free medium for additional 12-h culture. At endpoint, cells were collected and stained with Annexin V-FITC and propidium iodide, and then the percentage of apoptotic cells was determined by flow cytometry. The results are expressed as mean ± SD of the results of 3 independent experiments, each performed in triplicate. ** *P* < 0.01; *** *P* < 0.001.

Apoptosis and cell cycle arrest in cells stably transfected with miR-26a, miR-144, or both were analyzed via flow cytometry. The data revealed that co-expression of miR-26a and miR-144 in ESCC cell lines significantly induced both apoptosis and cell cycle arrest at G0 / G1 phase (Figure 2B, 2C and Table 1).

### MiR-26a and miR-144 inhibit migration and invasion of ESCC cells

Compared with the typical morphology of control cells, EC9706 and EC109 cells stably transfected with miR-26a, miR-144, or both were smaller in volume with a round-to-fusiform cell body (Figure 3A). This phenotype implied that miR-26a or mir-144 might affect metastasis of ESCC cells. Therefore, we undertook a further study of cell migration and invasion using a transwell chamber assay. The results showed that the migration and invasion abilities of ESCC cells stably transfected with miR-26a, or miR-144, or both were significantly suppressed, compared with the parent cells or vector-control cells (Figure 3B).

**Figure 3:** Ectopic expression of miR-26a, and miR-144, or both in ECC cells inhibited the metastasis ability of tumor cells **A.** Morphological changes in stably transfected cell lines and controls (×40). **B.** The metastasis ability (24 h) of tumor cells was determined by the assay using Matrigel-coated membrane to measure the amount of migrated cells. The results are expressed as mean ± standard deviation of data from 3 independent experiments, each performed in triplicate; *** *P* < 0.001.

### COX-2 was involved in the inhibitive effect of miR-26a and miR-144 on ESCC cells

To verify whether COX-2 is a target of miR-26a or miR-144 in human ESCC, we performed the following experiments. Firstly, the predicted binding sites of hsa-miR-26a and hsa-miR-144 in the 3′-UTR of COX2 mRNA is shown according to computational prediction, from which the luciferase reporters containing mutant binding sites were constructed (Figure 4A), to verify whether COX-2 is a direct target of miR-26a or miR-144 in human ESCC. The expression levels of miR-26a and miR-144 in EC9706 or EC109 stably transfected with miR-26a or miR-144 or both increased significantly (Figure 4B).

**Figure 4:** COX-2 expression is regulated by miR-26a and miR-144 in ESCC cells **A.** The predicted binding sites of hsa-miR-26a and has-miR-144 in the 3′ -UTR of COX-2 mRNA and their mutant counterparts. **B.** The expression levels of miR-26a or miR-144 in stably transfected ESCC cell lines. **C.** COX-2 expression in stably transfected cell lines was detected by western blot analysis as described in Materials and Methods. Beta-actin was used as an internal control to normalize COX-2 expression. **D.** Culture medium was collected for measurement of PGE2 levels using ELISA assay as described in Materials and Methods. **E.** Similar to protocol used in Figure 4B, the abilities of tumor cell invasion and migration in the presence of PGE2 were examined. Cells were cultured in serum-free medium supplemented with 40 μg / ml PGE2 for 24 hrs. **F.** Growth curve of the EC9706- miR-26a-144 cell line that was cultured in the medium supplemented with 40 μg / ml PGE2. **G.** 48 hrs after transfection of pMIR-COX-2-WT or pMIR-COX-2-MT, luciferase reporter activity was measured. Renilla luciferase was used for normalization. The data represent average value of triplicate samples from three independent experiments. ** *P* < 0.01; *** *P* < 0.001.

Secondly, we investigated the correlation of miR-26a or miR-144 with COX-2 expression in ESCC cells. Western blot analysis showed that overexpression of miR-26a, miR-144, or both in EC9706 and EC109 cells significantly reduced COX-2 expression at the protein level (Figure 4C). Furthermore, the level of PGE2, a primary product of COX-2 in stably transfected cells was significantly lower than that of parent and vector cells (Figure 4D; *P* < 0.001).

Thirdly, the inhibited proliferation of cells co-overexpression of miR-26a and miR-144 was promoted when PGE2 was added to the culture medium (Figure 4E; *P* < 0.001). Addition of PGE2 into the culture medium resulted in a significant increase in migration and invasion ability of cells stably transfected with miR-26a, or miR-144, or both (Figure 4F; *P* < 0.001).

Finally, to determine whether miR-26a or miR-144 can directly bind to the 3′-UTR of COX-2 mRNA, luciferase reporter activity of WT or MT pMIR-COX-2 plasmid in ESCC cells that overexpressed miR-26a or miR-144 was measured. Results showed that reporter activity of WT pMIR-COX-2 was significantly decreased in cells that over-expressed miR-26a or miR-144, as compared with the control cells (*P* < 0.01; Figure 4G).

### Co-expression of miR-26a and miR-144 potently inhibits the tumor formation and metastasis of ESCC *in vivo*

Co-expression of miR-26a and miR-144 in ESCC cell lines significantly inhibited the growth of xenograft tumors in nude mice, compared with mice inoculated with parental EC9706 or EC109 cells (Figure 5A).

**Figure 5:** Co-transfection of miR-26a and miR-144 inhibited both growth and metastasis of ESCC cells *in vivo* **A.** 1.5 × 10^6^ cells stably transfected with either vector or the combination of two miRNAs were implanted subcutaneously in both the right and left dorsal flank areas of nude mice (5 mice per group). Tumor volume was measured once a week over a period of 4 weeks. **B.** Nude mice were inoculated with 3 × 10^6^ cells by tail vein injection. Twelve weeks after inoculation, mice were killed and metastatic nodules on the surface of the livers were counted. In both (A) and (B), top panel displayed results of EC9706 groups, bottom panel for EC109 groups. *** *P* < 0.001.

The number of metastatic nodules on the surfaces of the liver was significantly less in mice inoculated single miRNA or two miRNAs-transfected ESCC cells than that of negative control mice (parent and vector groups), especially in the group with co-transfected miR-26a and miR-144 (Figure 5B, *P* < 0.001). No visible metastatic nodules on the lung, kidney, or spleen were found in either the miR-26a or miR-144 groups or in the control groups.

## DISCUSSION

In the present study, we investigated the effect of miR-26a and miR-144 on human ESCC. Firstly, we examined the expression levels of miR-26a and miR-144 in ESCC. A comparison between 30 pairs of ESCC tumor and adjacent normal tissues showed that the expression levels of miR-26a and miR-144 were significantly decreased in ESCC tumor (*P* < 0.001). Similar results were also found in 11 ESCC cell lines, suggesting that both miR-26a and miR-144 are downregulated in human ESCC. Secondly, we showed that miR-26a and miR-144 can reduce the migration and invasion abilities of ESCC cells. Co-expression of miR-26a and miR-144 in ESCC cells decreased cell proliferation by inducing apoptosis and cell cycle arrest at G0 / G1 phase. We further evaluated the inhibitory effect of miR-26a and miR-144 on ESCC using an *in vivo* study. Taken together, all of the data from the *in vitro* and *in vivo* studies indicated that miR-26a and miR-144 may function as tumor suppressors in ESCC. Thirdly, COX-2 as a direct target of miR-26a and miR-144 in ESCC cells was confirmed by means of luciferase reporter, western blot and ELISA. Our findings provide direct evidence to support that miR-26a and miR-144 are tumor suppressors in ESCC and inhibit ESCC by repressing COX-2 expression.

The involvement of miRNAs in the development and progression of ESCC has been reported in the literature [43–46]. Several miRNAs are upregulated and associated with tumorigenesis in ESCC, such as miR-21, miR-138, miR-223, miR-92a, miR-9, and mir-208. Aberrantly expressed miRNAs promote ESCC development through regulation of the expression of their target genes, such as PTEN (phosphatase and tensin homolog) and PDCD4 (programmed cell death 4), NF-κB, FBXW7 (F-box and WD repeat domain containing 7), E-cadherin and SOX6. On the other hand, some miRNAs are downregulated in ESCC, correlated with the loss of their function as tumor suppressors. For example, microRNA-375, miR-29c, miR-195, miR-625, miR-203, miR-302b, miR-133a, miR-101, miR-27a, miR-655 and miR-200b can suppress the growth of ESCC cells by regulating the expression of a variety of molecules, including IGF1R (insulin-like growth factor 1 receptor), cyclin E, Cdc42, Sox2, Ran, ErbB4, FSCN1 and MMP14, enhancer of zeste homolog 2 (EZH2), KRAS, ZEB1, TGFBR2 and Kindlin-2. In this study, we revealed the inhibitory effects of both miR-26a and miR-144 on proliferation and metastasis of ESCC.

The controversial functions of miR-26a and miR-144 in different types of cancers have been recently reported in the literature. MiR-26a can serve as tumor suppressor in many human cancers [47–59], but also as oncogene in cholangiocarcinoma [60], glioma [61–62], ovarian cancer [63] and T-cell acute lymphoblastic leukemia [64]. The role of miR-26a remains poorly defined in some cancers, because of conflicting reports. Some studies documented the anti-tumorigenic function of miR-26a in one type of cancer, but other studies found down-regulation of miR-26a in the same cancer type. Examples include lung [65–66], prostate [53, 67] and colon [68–70] cancers. Therefore, the roles of miR-26a in the progression of human cancer are poorly known.

The functions of miR-144 in human cancer development are also unclear. Although several reports showed that miR-144 is downregulated in hepatocellular carcinoma [71], non-small cell lung cancer [72], osteosarcoma [73], prostate cancer [74], cervical squamous cell carcinoma [75] and colorectal cancer [76–77], other studies showed that miR-144 can promote growth of HeLa cells [78] and cell proliferation, migration, and invasion in nasopharyngeal carcinoma [79].

The mature sequences of miR-26a and miR-144 are located at chromosomes 12q14.1 and 17q11.2, respectively. One of the common features of miR-26a and miR-144 is that both are located on chromosomal regions associated with various human cancers [80–82]. Another common feature of miR-26a and miR-144 is their discrepant functions in cancer development. For example, miR-26a inhibits growth of lung cancer cells by inhibiting EZH2 expression [65], but promotes lung cancer progression by suppressing PTEN [66]. Whether miR-26a is associated with lung cancer inhibition or promotion may depend on the protein level of EZH2 and PTEN in cancer cells. These present results suggest that miR-26a and miR-144 might be involved in the occurrence and development of cancer and the function of miR-26a and miR-144 in cancer is complicated and highly tissue-specific. This might be related with the different expression levels of different target genes. In this study, we selected EC9706 and EC109 cell lines as our model, because high COX-2 level in those cells was found in our previous study. In this study, we found that overexpression of miR-26a or miR-144 alone was not strong enough to inhibit proliferation of ESCC cells, but they still can inhibit COX-2 expression in cancer cells. This phenomenon might be associated with the differential regulation of downstream genes of COX-2 by these miRNAs. To clarify this hypothesis, further studies are needed. This phenomenon also reflects the complexity of miRNAs involved in tumorigenesis in the progression of various cancers.

Different miRNAs can bind to the same target mRNA to cooperatively block its translation [83], and this effect may be additive [84]. To clarify whether co-expression of miR-26a and miR-144 in ESCC cells has an additive effect, we constructed a special expression plasmid that can express both miR-26a and miR-144 simultaneously. In our study, ectopic expression of miR-26a or miR-144 alone in ESCC cells was not strong enough to inhibit tumor growth, while co-expression of both miR-26a and miR-144 led to the inhibition of ESCC cell proliferation and stronger suppression of ESCC metastasis, compared with the similar effects of the individual miRNAs. This suggests that there is an additive inhibitory effect by the co-expressed miR-26a and miR-144 on COX-2 expression and cell proliferation and metastasis in ESCC.

Recent progress in delivery technology of tumor-suppressive miRNAs offers the possibility of promising new approaches to treat cancer. Among miRNA-based approaches using an *in vivo* delivery system with DNA plasmids or viral vectors, miRNA replacement therapy with double-stranded RNAs mimicking miRNAs may be one of the most promising [85–87]. Since COX-2 is considered a potential therapeutic target of ESCC, our findings suggest that miR-26a and miR-144 may contribute to a novel therapeutic approach for ESCC.

In conclusion, expression of miR-26a and miR-144 is downregulated in cell lines and tumor tissue specimens of ESCC. In our *in vitro* and *in vivo* studies, co-expression of both miR-26a and miR-144 in ESCC resulted in the inhibition of either proliferation or metastasis. COX-2 is confirmed as a direct target of miR-26a or miR-144, and inhibition of COX-2 expression might be the action mechanism underlying their anti-tumor functions.

## MATERIALS AND METHODS

### Ethics statement

The Clinical Research Ethics Committee of Beijing Friendship Hospital, Capital Medical University approved the project and protocol for the investigations involving humans and animals. The study was thus performed in accordance with the ethical standards laid down in the Declaration of Helsinki. All participants provided their written informed consent to participate in this study, and the ethics committee approved this consent procedure.

### Collection of ESCC clinical samples and culture of ESCC cell lines

Thirty pairs of primary esophageal squamous cell cancer tissues and corresponding adjacent normal esophageal tissues were obtained from untreated patients in Beijing Friendship Hospital (Capital Medical University) from 2009 to 2011 with informed consent and agreement. All tissue samples were snap frozen in liquid nitrogen and stored at −80°C until the extraction of RNA.

The human ESCC cell lines KYSE30, KYSE70, KYSE150, KYSE410, KYSE450, KYSE510, EC9706, and EC109 were kindly provided by the Cancer Institute and Hospital, Chinese Academy of Medical Science. The ESCC cell lines TE-1, TE-9, and TE-11 were gifts from Hebei Cancer Hospital of China. Het-1A, a human esophageal immortalized cell line, was purchased from the American Type Culture Collection. Five-week-old male BALB/c nu/nu mice were purchased from the Institute of Laboratory Animal Sciences, Chinese Academy of Medical Sciences. ESCC cell lines used in this study are listed in previous reports [14-15, 88-90].

All cell lines, except for Het-1A, were cultured in RPMI-1640 medium (Hyclone, USA) containing 10% fetal bovine serum (Gibco, USA) and 10 units / ml penicillin and streptomycin (Hyclone, USA). Cells were maintained at 37°C, 95% humidity, and 5% CO_2_. Het-1A cells were cultured in bronchial epithelial basal medium with growth supplements (Clonetics, USA).

### Real-time quantitative reverse-transcription (RT)-PCR

To measure the expression levels of mature miR-26a and miR-144, real-time quantitative RT-PCR was performed as previously described [48]. The miRNAs were extracted from cultured cells or frozen tissues with a mirVana miRNA Isolation Kit (Applied Biosystems, USA). Ten nanograms of the extracted miRNAs were reverse-transcribed to cDNA using a TaqMan MicroRNA Reverse Transcription Kit (Applied Biosystems, USA). The reaction mixture was used for real-time RT-PCR of miR-26a and miR-144, using an Applied Biosystems 7500 Fast System and standard TaqMan PCR reagents. U6 was used as an internal control. Fold changes for the expression levels of miR-26a and miR-144 were calculated using the comparative cycle threshold (CT) method (2^−ΔΔCT^). All miRNA samples were run in triplicate in real-time quantitative RT-PCR.

### Construction of expression plasmids and selection of stable clones

The specific primers for establishing expression plasmids of miR-26a and miR-144 were:

miR-26a, sense 5′-CG G / GATCC (*Bam*HI) TGACTGTAAGCATGACTGGCCTG-3′;

miR-26a, anti-sense 5′-CTACATGCAAAGG GCAGGAGA A / AGCTT (*Hind*III) GGG-3′;

miR-144, sense 5′-CG G / GATCC (*Bam*HI) TCACAGTGCTTTTCAAGCCATG-3′; miR-144,

anti-sense 5′-CAAGTGCCCTGGCAGTC AGTA A / AGCTT (*Hind*III) GGG-3′. (Restriction sites were underlined in each primer.)

Precursors of miR-26a (351 bp) and miR-144 (220 bp) were cloned into the pSilencer 4.1-CMV vector (Ambion, Geneworks), in accordance with the manufacturer's instructions. The expression plasmid for the miR-26a-144 cluster was made in three steps: 1) An integrated plasmid of miR-26a and miR-144 was prepared by PCR (miR-26a, 368 bp; miR-144, 236 bp) with primers: miR-26a, sense 5′-GC T / CTAGA (*XBa*I) TGACTGTAAGCATGACTGGCCTG-3′; miR-26a, anti-sense 5′-TCTCC TGCCCTTTGCA TGTAG A / AGCTT (*Hind*III) GGG-3′; miR-144 sense, 5′-CG G / GATCC (*Bam*HI) TCACAGTGCTTTTCAAGCCATG-3′; miR-144, anti-sense TACTGACTGCCAGGGCAC TTGG T / CTAGA GC (*XBa*I)-3′. 2) Two PCR fragments were digested by *XBa*I and then connected to each other to form a longer fragment that included 5′-*Bam*HI and 3′-*Hind*III sites and protective bases. 3) A larger DNA fragment (594 bp) was amplified, cut by *Bam*HI and *Hind*III, and inserted into the pSilencer 4.1-CMV vector.

Introduction of the expression plasmids carrying miR-26a, miR-144, and miR-26a-144 into EC9706 and EC109 cells was performed using Lipofectamine 2000 (Invitrogen, USA) in accordance with the manufacturer's instructions. Stably expressed cell lines were selected with G418 (Sigma, USA) at dose of 600 mg / ml and maintained at 300 mg / ml. The expression levels of miR-26a and miR-144 in stable clones were verified via real-time RT-PCR.

### Cell proliferation assay

Cell proliferation was measured with a Cell Counting Kit-8 (CCK-8, Dojindo, Japan). Colorimetric assay and growth curves were created using the mean results from three independent experiments. Briefly, cells were seeded at density of 5 × 10^3^ cells per well in a 96-well plate. Cell viability was assessed using the Cell Counting Kit at 24, 48, 72, 96, and 120 h after transfection. The absorbance at 450 nm was measured with a plate reader.

### Cell cycle analysis and detection of apoptosis

Dissociated cells were fixed and permeabilized with cold 70% ethanol, overnight at 4°C. The next day, cells were stained with 10 μL of 1 mg / ml propidium iodide and 10 μl of 500 μg / ml RNase (37°C for 30 min) for flow cytometry. Cells stained with Annexin V-FITC and propidium iodide were used for determining the rate of apoptosis by flow cytometry, in accordance with the protocol of the FITC Annexin V Apoptosis Detection Kit I (BD Pharmingen, USA).

### Cell migration and invasion assays

The capability of cell migration and invasion (incubation for 24 h) were analyzed using non-Matrigel-coated (BD Falcon cell culture inserts, BD Biosciences, USA) or Matrigel-coated transwell cell culture chambers (BD Matrigel Invasion Chamber, BD Biosciences, USA), of 8 μm pore size, in accordance with the manufacturer's instruction.

### Western blot

Western blot analysis was performed as described in our previous publication [14]. The primary antibodies and secondary antibody used in this study were rabbit anti-COX-2 antibody (1:1000, Cell Signaling, USA), rabbit anti-β-actin antibody (1:1000, Sigma, USA), and sheep anti-rabbit antibody conjugated to horseradish peroxidase (1:6000, Santa Cruz, USA).

### Dual-luciferase reporter assay

Luciferase reporters of COX-2 were made through RT-PCR using the following primers:

(1) WT-binding sites of miR-144 (490 bp), upstream primer with a *Sac*I site (5′-GCCACAGAGCT / C AGCTATCTGTAACCAAGATGGATGC-3′) and downstream primer with a *Hind*III site (3′-GTCCTTAGGATAGGCCTATGTGCTA A / A GCT TCCGCAT-5′);

(2) wt-binding sites of miR-26a (300 bp), upstream primer with a *Sac*I site (5′-GCCACAGAGCT / C ACAGAAGTCAGTACTCCTGTTGC-3′) and downstream primer with a *Hind*III site (5′-CTTCTAATGC ATCATGGAAG ATGC A / AGCTT CCGCAT-3′).

Luciferase reporters of COX-2 with mutant binding sites (underlined and italicized) of miR-26a or miR-144 were made using two DNA fragments with 5′ *Sac*I and 3′ *Hind*III sites (underlined) and protective bases. Shown below, each was synthesized by Sangon Biotech (Shanhai). A mutant of the miR-144 binding site (144 bp): GCCACA GAGCT / CAATAATAATGACGATAATACTTCTTTTCCACATCTCATTGTCACTGACATTTAATGGAC*GGT*TATATTACTTAATTTATTGAAGATTATTATTTATGTCTTATTAGGACACTATGGTTATA / AGCTTCCGCAT; and a mutant miR-26a binding site (144 bp): GCCACAGAGCT / CTTAAGTTTGGAAAACAGTTTTT ATTCT GTTTT ATAAACCAGAGAGAAATGAGTTTTGACGTCTTTT*CGTGCC*AATTTCAACTTATATTATAAGAACGAAAGTAAAGATGTTTGAATACTTA / AGCTT CCGCAT.

PCR products or synthetic DNA fragments were digested and cloned into *Sac*I and *Hind*III sites on a pMIR-REPORT miRNA Expression Reporter Vector (Ambion, USA), finally confirmed by DNA sequencing.

To perform a luciferase reporter assay, EC9706-miR-26a or EC9706-miR-144 cells (4 × 10^4^) were seeded in a 48-well plate and then co-transfected with 800 ng of reporter of either wild type (WT) (pMIR-miR-26a WT or pMIR-miR-144 WT) or mutant type (MT) (pMIR-miR-26a MT or pMIR-miR-144 MT) or 40 ng of pMIR-vector and 4 ng of pRL-TK vector (Promega), an internal control using Lipofectamine 2000 (Invitrogen). Forty-eight hours after transfection, cells were collected for analysis using a Dual-Luciferase Reporter Assay Kit (Promega), in accordance with the manufacturer's instructions. Results were measured with a GloMax-Multi Detection System (Promega). Transfection was done in duplicates and experiments were repeated at least thrice.

### Tumor formation in nude mice

Stably transfected cells (1.5 × 10^6^ in 0.2 ml) were injected subcutaneously into the right (EC9706-miR26a-144 or EC109-miR26a-144) and left (EC9706-vector or EC109-vector) dorsal flank of 5-week-old severe combined immunodeficiency (SCID) mice (Institute of Laboratory Animal Sciences, Chinese Academy of Medical Sciences), five mice per group. Tumor size was determined by the formula volume = 0.5 × length × W^2^, at 4-week after inoculation of tumor cells.

### Metastasis assay in nude mice

Stably transfected cells were injected intravenously (3 × 10^5^ per mouse) into 5-week-old SCID mice through the tail vein. There were two groups (EC9706-vector or EC109 and EC9706-miR26a-144 or EC109-miR26a-144) in animal study and each group had five mice. The number of tumor nodules formed on the surface of the liver, lungs, kidney and spleen was counted at 12- week after injection.

### Enzyme immunoassay for prostaglandin E2 (PGE2)

PGE2 in the culture supernatant was measured by enzyme-linked immunosorbent assay (ELISA), in accordance with kit manufacturer's protocol. The concentration of PGE2 was expressed as picograms per milliliter.

### Statistical analysis

SPSS 15.0 software (Chicago, IL, USA) was used for statistical analysis in this study. Data were presented as means ± SD, which were collected from at least 3 independent experiments. Two-tailed Student's t-test was used for comparisons of two independent groups. *P* < 0.05 was considered statistically significant.
